The article "Risk Analysis of A-H Share Connect Market Based on Deep Learning and BP Neural Network" was published in 2022. Journal: Comput Intell Neurosci.

# Risk Analysis of A-H Share Connect Market Based on Deep Learning and BP Neural Network

**DOI:** 10.1155/2022/1921463

**Published:** 2022-07-21

**Authors:** Rumeng Cui, Wen Chen

**Affiliations:** School of Economics and Management, Beijing Jiaotong University, Beijing 100044, China

## Abstract

China's Shanghai-Hong Kong Stock Connect and Shenzhen-Hong Kong Stock Connect programs make it possible for investors to trade stocks within specified limits through the two stock exchanges. The A-H share exchange stock market is crucial to the opening of the Mainland market, but few studies have paid attention to the market risks of such stocks. Using deep learning and BP neural network algorithm, this study constructs a three-dimensional A-H share interconnection market risk prediction index system including stock price fundamental indicators, technical indicators, and macro indicators based on the CES300 Index. Taking the CES300 Index return as the output layer indicator, a BP neural network with a 21-10-1 structure is constructed, and the tan-sigmoid transfer function and the LM optimization algorithm training function are used for network training to predict the return of the A-H share interconnected stock market. The mean square error (MSE) converges to 10^−6^, and the goodness of fit *R* reaches 0.9928 and validates the prediction accuracy of the BP neural network model. It provides an efficient and accurate risk prediction model for the A-H share interconnected market, which facilitates the interactive development of the Mainland and Hong Kong markets.

## 1. Introduction

The Shanghai-Hong Kong Stock Connect was launched in November 2014, which established a technical channel between the Shanghai Stock Exchange and the Hong Kong Stock Exchange. This allows investors to trade some of the shares listed on the counterparty's exchange through the local stock exchange. Subsequently, the Shenzhen-Hong Kong Stock Connect was launched in 2016, which help to open up two Mainland markets. Equity market risk is the risk of not being as profitable as investors expect due to fluctuations in market prices. As an emerging stock market, China's capital market usually faces higher risks due to its immature investors, unsound market mechanism, and excessive growth rate (Kohers et al.) [1]. This exchange policy has increased the risk correlation between the two markets. However, few researchers care about the interconnection between the Mainland stock market (A-share) and Hong Kong stock market (H-share) (Liu and Kemp; Li and Bastos) [2, 3].

The stock market is a highly complex nonlinear dynamic system, and many factors may affect the fluctuation of this nonlinear dynamic system. The development of computer technology makes it possible to anticipate market risks. Deep learning based on back-propagation neural network (BPNN) learns more useful features by building a machine learning model with many hidden layers and massive training data, thereby ultimately improving the accuracy of classification or prediction. As an efficient information processing algorithm, BP neural network can model the inherent relationship of data and has a good comprehensive ability to deal with chaotic data. The existing research shows that the three-layer BP neural network is the best for predicting nonlinear functions. The BP neural network is properly adjusted to handle any nonlinear problem until the specified accuracy is achieved. Therefore, this study utilizes the BPNN algorithm to predict the A-H connect stock market risk, it can be used to track changing stock prices, and based on this, investors can judge the timing of investment and reduce investment risks.

The article "Risk Analysis of A-H Share Connect Market Based on Deep Learning and BP Neural Network" was published in 2022. Journal: Comput Intell Neurosci.

The stock price index can accurately and comprehensively reflect the fluctuations and changes of the stock market and is an important indicator of market risk prediction. Based on the stock index CES300, this study comprehensively considers the price fluctuation of the A-H share exchange market, establishes a risk prediction index system, and uses BP neural network to build a prediction model for market risk analysis. The innovation of this exploration lies in the following two aspects: (1) based on the A-H connect stock index, combined with micro transaction data and macroeconomic data, the risk prediction index system of the A-H stock connect market is constructed. At present, there is no research focusing on the risk forecast of the stock market formed under the Shanghai-Hong Kong Stock Connect policy. (2) Through the application of deep learning and BP neural network, the optimal parameters are adjusted by testing, and the optimal fitting model is constructed, which verifies the accuracy and feasibility of the BP neural network in predicting the market risk of A-H connect stock. This study expands the method of stock market risk prediction formed by the Shanghai-Hong Kong Stock Connect policy.

The research arrangement of this study is as follows: Section 2 presents the related literature.  Section 3 demonstrates the principles of model design and BPNN parameter setting, and according to indicators of market risk, the risk assessment model is constructed.  Section 4 carries out network training and analysis of training results.  Section 5 uses new test data to further determine the validity of the model and conduct market risk analysis.  Section 6 offers conclusions and limitations of research.

The article "Risk Analysis of A-H Share Connect Market Based on Deep Learning and BP Neural Network" was published in 2022. Journal: Comput Intell Neurosci.

## 2. Literature Review

The operation of the stock market is affected by other factors besides macroeconomic and microeconomic factors. The models used to predict stock prices can be roughly divided into three views: the first is based on the efficient market hypothesis and the stochastic volatility hypothesis, which believes that investors cannot obtain returns that exceed the level of the securities market based on current and historical data; the second view is that macroeconomics. There is a corresponding fluctuation relationship between the microeconomic factors, the financial situation of the enterprise, and the fluctuation of the stock price; the third believes that a mathematical model needs to be established to predict the stock market.

In the above three viewpoints, scholars have adopted different methods to analyze. The traditional statistical method includes moving smoothing, exponential smoothing, regression, ARIMA, and GARCH models. Engle (1982) proposed the ARCH model and added random disturbance terms to solve the problem that the time series model cannot well decompose the fluctuation of financial time series fluctuations with time [4]. Bollerslev proposed the GARCH model and introduced the time-varying variance of financial asset prices [5]. Jiang and Subramanian took the U.S. stock market as the research object and proposed an autoregressive comprehensive average model to predict the value of future stocks [6]. However, traditional statistical forecasting has shortcomings such as prediction lag, large noise, and high correlation of influencing variables. In recent years, various algorithms and machine learning have been used by scholars to predict financial markets (Shah et al.; Picasso et al.; Ramezanian et al.; Harel and Harpaz) [7–10]. Honchar and Di Persio used the price data of the S&P 500 Index to establish MLP, CNN, and RNN models, respectively, and used the closing price to predict the rise and fall of the next day [11]. Hochreiter and Schmidhuber proposed the RNN variant neural network model, namely, long short-term memory (LSTM) network, which can well solve the problems of gradient disappearance and gradient explosion [12].

Ergezinger and Thomsen pointed out some shortcomings, and the neural network is prone to the problem of local minima, the problem of premature convergence, and so on [13]. In this case, in order to solve some of the above problems, Sexton et al. used the global search technique to optimize the weights and thresholds of the BP neural network [14]. BP neural network just makes up for this shortcoming, and existing studies have used empirical tests and found that BPNN can indeed predict trends more accurately and reduce errors (Fang et al.) [15]. Existing research utilized the BPNN algorithm to predict monetary policy (Lu) [16], stock price (Huo et al.) [17], Internet financial risk (Qi et al.) [18], supply chain financing risk (Cai et al.) [19], and *A* + *H*-share price (Wu et al.) [20], but no one used to predict the market risk of A-H connect stock market.

The article "Risk Analysis of A-H Share Connect Market Based on Deep Learning and BP Neural Network" was published in 2022. Journal: Comput Intell Neurosci.

## 3. BP Neural Network Model Design

The BP neural network is established based on the information transmission model of human brain neurons. It belongs to a multilayer feedforward neural network, which can forward the information at the input and reversely adjust the information with errors. In order to achieve the accuracy, set by the BP neural network, the BP neural network will actively and continuously adjust the thresholds and weights between each level. The BP neural network consists of three parts: the input layer, the hidden layer, and the output layer. Each layer involves a large number of neurons, and these three layers are also organically combined by these neurons to form the integrity of the model. Continuous training is performed by sample data collected in advance, and the program debugs the number of nodes in the hidden layer of the BP neural network (BPNN) and the input layer data to modify the weights and thresholds of the network, so as to achieve the goal of reducing the error function along the negative gradient direction and finally get the desired output.

Figure 1 depicts the basic architecture of BPNN selected in this study. We mainly use a three-layer neural network, which in short means that only one layer of neurons (called the hidden layer) exists between the input and output layers. In this structure, changes in the state of the middle hidden layer can affect the relationship between the input and output layers, although it is not directly linked to the external data, and in addition, each layer in the neural network can have multiple nodes. In our deep learning training procedure, the set input layer nodes are linked to market risk indicators, while the output layer nodes are set with only one node as the index return.

The main parameter design of BPNN includes input layer nodes, output layer nodes, transfer function, hidden layer nodes, learning rate, and training function. This section mainly introduces the design of neural network parameters and the construction of the index system.

### 3.1. Input Layer and Output Layer Index System

#### 3.1.1. Input Layer: Market Risk Prediction Indicator System

This study selects the CES300 Index (CES105.CSI) as the basis for the construction of the index system. China 300 Index is a comprehensive stock index provided by China Securities Index Co., Ltd. that reflects the overall trend of the connected stock market between Mainland and Hong Kong, including 100 stocks with the largest market capitalization in Shanghai-Hong Kong Stock Connect, Shenzhen-Hong Kong Stock Connect, and Hong Kong Stock Connect. The index accounts for 61% of the total market value of stocks with A-H share interconnection qualifications and 38% of the total market value of the connected stock market between Mainland and Hong Kong. CES300 was launched on 2014-12-15, the base period for index calculation was 2008-12-31, and the base point of the index was 2000.

The article "Risk Analysis of A-H Share Connect Market Based on Deep Learning and BP Neural Network" was published in 2022. Journal: Comput Intell Neurosci.

At the market level, stock price fluctuations are affected by micro and macro factors. This study constructs an index system that affects stock returns from three dimensions for risk analysis.

First, the data variables of fundamentals include “opening price,” “closing price,” “highest price,” “lowest price,” “trading volume,” and “trading value” which is based on the CES300 Index. It reflects the basic trading conditions and stock price levels of the interconnected markets of the three stock exchanges.

Second, micro-expanded data variables include “P/E,” “P/B,” and “P/E change rates,” in which the “P/B change rate” is derived from the China 300 Index. At the same time, the interval data are expanded for the variables, and dynamic change data of stock data are added, such as “volatility 20 days,” “volatility 60 days,” “volatility 120 days,” and “volatility 250 days,” reflecting how the closing price has fluctuated over the past few days. The formula for calculating these indicators is as follows:

(1) $$\begin{array}{c} \sigma_{x}=\sqrt{\frac{\sum_{i=1}^{n}{\left(x_{i}-\mu_{x}\right)}^{2}}{n-1}}. \end{array}$$

In the above equation, *n* represents the time interval, which are 20, 60, 120, and 250, respectively. *x*_*i*_ and *μ*_x_ represent the logarithmic rate of return and the average rate of return in the interval, respectively.

In addition, the technical indicator data variables, including the deviation ratio (BIAS) (BIAS is the standard code for the deviation ratio in Chinese stock trading software), in equation (2), and moving averages (MA), in equation (3), are introduced.

BIAS is a measure of how much a stock price deviates from the moving average. It reflects the likelihood of a pullback or rebound in the stock price when the price moves significantly, with pullbacks and rebound originating from deviations from the moving average trend. It also implies the plausibility of a stock closing price adjustment back to its original trend within the normal range of volatility, as shown in the following equation:

(2) $$\begin{array}{c} \text{BIAS}=\frac{{\text{CP}}_{i}-\left(1/n\right)\sum_{i=1}^{n}{\text{CP}}_{i}}{\left(1/n\right)\sum_{i=1}^{n}{\text{CP}}_{i}}\times 100\%, \end{array}$$

where CP is the closing price. In this study, *n* = 6 is set, that is, the deviation of the closing price within 6 days.

The article "Risk Analysis of A-H Share Connect Market Based on Deep Learning and BP Neural Network" was published in 2022. Journal: Comput Intell Neurosci.

MA can more intuitively show the past fluctuations of the stock and objectively reflect the state of the stock market. The moving average theory helps investors to confirm the current trend of the stock and judge the trend that will appear and reverse. The calculation formula is as follows:

(3) $$\begin{array}{c} \text{MA}=\frac{\sum_{i=1}^{n}{\text{CP}}_{i}}{n}, \end{array}$$

where CP is the closing price. In this study, *n* = 14 is taken, which is the moving average of the stock price volatility in the past 14 days.

Third, macro impact indicators. The A-share and H-share interconnection markets will also be affected by macro-influencing factors such as economy and politics. In this study, the following indicators of macroeconomic factors are included in order to provide a comprehensive picture of the external economic environment on the stock market, in particular, the exchange rate of US dollar (day), Hong Kong dollar exchange rate (day), CPI year-on-year (month), M2 year-on-year (month), and GDP (quarter).

The exchange rate risk triggered by the A-H stock exchange can be divided into three levels: first, investors need to bear exchange rate risk regardless of bookkeeping mode or foreign exchange mode; second, in the exchange mode, large settlement and sales will also impact the market exchange rate; third is the reverse effect of exchange rate fluctuations on the relevant stock market. In the foreign exchange market, the Hong Kong dollar is pegged to the U.S. dollar and fluctuates only within a narrow range. Obviously, the exchange rate risk of the RMB to the Hong Kong dollar is equivalent to the risk of the RMB to the U.S. dollar. In short, when the US dollar depreciates, the exchange rate of Hong Kong dollar also falls. Therefore, this study includes exchange rate indicators USD exchange rate (daily) and HKD exchange rate (daily).

M2 is a common indicator of the money supply, which indicates the cash circulating outside a country's banking system and, when added to corporate deposits, savings deposits of the country's residents, and other deposits, mainly implies the money circulating freely in the capital markets. If M2 growth represents an increase in the money in circulation in the market, then more money will flow into the stock market.

GDP is the total value of all products and services expressed in money within a country during a certain period of time. A rise in GDP indicates strong economic growth and can increase consumer confidence. At this time, the enthusiasm for participating in stock market investment is also very high, which can stimulate stock market development and push up stock prices.

The article "Risk Analysis of A-H Share Connect Market Based on Deep Learning and BP Neural Network" was published in 2022. Journal: Comput Intell Neurosci.

The CPI affects the stock market's rise and fall through the supply and demand relationship on the capital side. When monetary policy is looser and risk-free interest rates are low, the stock market will attract liquidity funds to enter and then pull up the stock index. However, stock indexes cannot keep rising. In the case of excess liquidity in the capital market, as a result of experience, CPI will continue to rise, at which time the state will certainly introduce stricter monetary macro-control policies. Along with that, if the reserve ratio and interest rate of commercial banks increase, then the enthusiasm of deposits will be higher than the tendency to invest in the stock market, and the capital market liquidity will decrease, which will indirectly lead to changes in the stock index.

#### 3.1.2. Output Layer: The CES300 Index Return

This study uses the return rate of the CES300 Index on the next day as the output layer of BPNN to reflect the overall return of the A-share and B-share interconnection market, as shown in the following equation:

(4) $$\begin{array}{c} {\text{DY}}_{t}=\frac{\text{Closing }{\text{Price}}_{t}-\text{Closing }{\text{Price}}_{t-1}}{\text{Closing }{\text{Price}}_{t}}, \end{array}$$

where DY is the return rate of the CES300 Index, *ClosingPrice*_*t*_ represents the closing price of the CES300 Index on trading day *t*, and *ClosingPrice*_*t*−1_ represents the closing price with a one-day lag.

Figure 2 shows the volatility of CES300 Index yields from January 2015 to the end of 2021. The highest point of yield occurred in July 2015, and the lowest point was in August 2015. The index yield fluctuates greatly and has a certain periodicity. The yield volatility of the China 300 Index has narrowed year by year, along with the deepening of the policy of interconnection of securities trading between Mainland China and Hong Kong. Predicting the volatility of the CES300 index can provide a basis for observing the market risk of the A-H connect market.

### 3.2. Transfer Function

A transfer function, also called an activation function, is needed to eliminate the effect of the difference in size of different data on the training results. The data are normalized by the transfer function and then passed from the input layer to the hidden layer of the BPNN. The training efficiency of BPNN can be affected by different choices of transfer functions. There are many transfer functions of BPNN. Linear transfer function (purelin) can have arbitrary input and output values; tan-sigmoid transfer function (tansig) can have arbitrary input values and output values in the range of [−1, 1]; log-sigmoid transfer function (logsig) can have arbitrary input values and output values in the range of [0, 1]. Considering the training efficiency and the positive and negative values of the output variable data type selected in this study, this study uses the tan-sigmoid function, which means that the real value range of the hidden layer output is [−1, 1], and its expression is as follows:

(5) $$\begin{array}{c} f\left(x\right)=\frac{1-e^{-x}}{1+e^{-x}}. \end{array}$$

In this study, the raw data of each indicator in Table 1 are normalized as described above, and the processed data are used as information in the input layer of BPNN. The same transformation is done for the output layer data.

The article "Risk Analysis of A-H Share Connect Market Based on Deep Learning and BP Neural Network" was published in 2022. Journal: Comput Intell Neurosci.

### 3.3. Hidden Layer Nodes

The number of input layer nodes in the BPNN model in this study is 21, which is equivalent to the number of indicators in the risk analysis index system. The hidden layer of the BP neural network should not be too many; otherwise, the model test time will be greatly increased, resulting in the smallest local error and failure to converge. In practice, two-layer network learning is usually performed. Regarding how to choose the number of nodes in the hidden layer, we can follow the Kolmogorov theorem to find the answer. Specifically, the following equation is used to obtain the range of values, and then, the number in this range of values is tested one by one and selected on merit:

(6) $$\begin{array}{c} H=\sqrt{m+n}+a. \end{array}$$

In the above equation, H represents the number of nodes in the hidden layer, *m* + *n* represents the sum of the number of nodes in the input and output layers, and a is a regulation constant between 1 and 10. In the specific context of this study, the input layer nodes *m* = 21 and output layer nodes *n* = 1 are substituted in equation (6) to obtain the lower threshold 5. After adding the constant a, we calculate that the optimal number of nodes in the hidden layer falls in a range of [5, 15], so we need to test them one by one in this value interval. After several rounds of testing one by one, the best fitting effect occurs when the number of nodes in the hidden layer takes the value of 10.

In summary, a BPNN model with a 21-10-1 type structure is established in this study and presented in Figure 3. As shown in Figure 3, the essence of neural network learning is to use the loss function to update the weight parameter *w* iteratively to achieve better performance. The nodes in the input layer are 21, the nodes in the hidden layer are 10, and the nodes in the output layer are 1. In the input and output layers, where *w* represents the weight parameter and *b* represents the bias can be shifted up or down to better fit the prediction to the data.

The article "Risk Analysis of A-H Share Connect Market Based on Deep Learning and BP Neural Network" was published in 2022. Journal: Comput Intell Neurosci.

## 4. Network Training and Testing Results

This section mainly introduces the neural network training process, selects the training function and training judgment criteria, and finally obtains the model validity.

Next, the training process of the BP neural network in this study is described, as shown in Figure 4:

 
*Initialize the Network*. Design the input layer and output layer design, divide the data set, normalize the data, set the error function e, and set the learning rate and the maximum number of learning.
 
*Calculate the Error*. The *n*th training sample is randomly selected and the input and output of each node in the hidden layer are calculated; calculate the bias derivatives of the error function for each node in the output layer based on the expected output and the actual output of the network; use the bias derivatives of the nodes in the output layer and the output of each node in the hidden layer to correct the link weights; use the bias derivatives of the nodes in the hidden layer and the data in the input layer to correct the link weights; recalculate the global error of the new model.
 
*Judge the Model Validity*. In other words, judge whether the current model meets the error convergence requirement and the best-fit merit; otherwise, select the next random training sample and the corresponding expected output and perform the next learning.

The network training data in this study come from the stock index database in the Oriental Fortune website, as well as the macroeconomic database. The MATLAB software was used for model fitting. The data sample period was from January 2, 2015, to December 31, 2021. Missing data were excluded. There were 1744 groups of historical data, and the data were in daily units. About 70% of the training set, 15% of the validation set, and 15% of the test set constitute the training data initialized in this study. The data on the training set train the model and generate model parameters. Then, the optimal parameters of the model are selected on the validation set. Finally, the test set is used to test the effects of the current network.

In the study of BP neural networks, trainlm, trainingdx, and traingd are commonly used training functions by scholars. This article uses trainlm, the LM (Levenberg–Marquardt) optimization algorithm. For medium-sized networks, the LM optimization algorithm is the fastest to train but has the disadvantage of taking up a lot of memory. Due to the small size of the network in this study, the LM optimization algorithm is selected for training.

The article "Risk Analysis of A-H Share Connect Market Based on Deep Learning and BP Neural Network" was published in 2022. Journal: Comput Intell Neurosci.

Meanwhile, the effectiveness of the network training model is evaluated using MSE (mean squared error). The learning algorithm adopts the common elastic gradient descent method. MSE is calculated as follows:

(7) $$\begin{array}{c} \text{MSE}=\frac{1}{n}\sum_{i=1}^{m}{\left(f_{i}-y_{i}\right)}^{2}, \end{array}$$

where *y*_*i*_ represents the expected *i*th output value of the neural network and *f*_*i*_ indicates the actual output value. *n* corresponds to the number of samples in the data set. The error standard set in this study is *ε* = 0.001.

The choice of learning rate will affect the network training time and the speed of error convergence. When the learning rate is set too low, the network training time becomes longer, and the convergence rate slows down; conversely, the learning rate is too high and will start to diverge before reaching the desired accuracy error range. In our tests, the learning rate was set to *η* = 0.01, while the maximum number of learning times was chosen to be 1000. Ultimately, we judge the reasonableness of the learning rate setting by observing the rate of decline of the error curve, which is obtained by network training.

Based on the previous settings, the system converges to the error criterion at a very fast rate through iterative learning and training to obtain the optimal prediction value.  Table 2 lists the training results. As shown in Figure 5, the best validation performance is 1.2718e-05 at epoch 19, and the convergence speed is fast. After learning and training from Figure 6, the error of fitting the three datasets is small, and it is concentrated around 0.

After deep learning through the BP neural network, the goodness of fit of each group of data sets can be obtained. The four bars in Figure 7 reflect the effect of fitting the data in different data sets. Among them, the goodness of fit *R* of the training sets is 0.9928, and the goodness of fit of the validation set is 0.95395. The goodness of fit of the test set is 0.94288 and the goodness of fit of all data sets is 0.99003. The degree *R* converges to 1, which proves that the network training effect is excellent.

With the above settings, investors can collect data from the new indicator system and recalculate the output layer of the network model based on the training results, thus predicting market return trends and providing a data base for market risk analysis.

## 5. Model Retesting and Market Risk Analysis

In the network training phase, due to the randomness of the test set, this study uses a new dataset to verify the prediction accuracy of the constructed network model again. We select the data from January 1, 2021, to February 4, 2022, as a new test set to fit the exponential returns of the past year. The training results show that the goodness of fit *R* is 0.95, and the error converges to 10^−6^. The validity of the model is checked again, and the risk analysis of the A-H share interconnection market is carried out. The new test sample data are substituted into the network model, and the actual and expected outputs are presented simultaneously in Figure 8.

The article "Risk Analysis of A-H Share Connect Market Based on Deep Learning and BP Neural Network" was published in 2022. Journal: Comput Intell Neurosci.

Figure 8 depicts the gap between the true and fitted values, and the results in the figure corroborate the high prediction accuracy of our constructed BPNN model. According to the yield trend in the figure, the yields of the A-H share interconnection market have fluctuated greatly and frequently in the 277 trading days in the past year. In early 2021 and mid-2021, there will be large fluctuations, and the latter will show a state of shock and convergence. The peak occurred in mid-2021 and was negative, −4.7%. The figure shows that market yield fluctuations are cyclical. With the deepening of the interconnection policy between Hong Kong and Mainland stock markets, the volatility of the CES300 index has been narrowing.

## 6. Conclusions

Stock market risk has a long history and is a universal problem worldwide. The interconnection between the Mainland and the Hong Kong stock exchange has brought vitality to A shares and H shares, but also added new market risks. In view of deep learning and BPNN technology, this research utilizes relevant data of the CES300 Index to construct the A-H share interconnection stock market risk prediction index system and adopts a reasonable selection of experimental parameters to establish a training model and a test model. A BP neural network model with a 21-10-1 structure was established using MATLAB and the hardware has no special needs and is completed using only a Windows-based computer. Finally, the effectiveness of our model in the risk assessment process of A-H share interconnected market is trained and tested, and it is verified that the BPNN method is effective in the construction of the A-H share interconnection market risk assessment model.

Based on fundamental indicators, micro-expansion indicators, and macro-influencing indicators, this study conducts risk analysis on the A-H share connect market. The development of Shenzhen-Hong Kong Stock Connect and Shanghai-Hong Kong Stock Connect has increased the linkage between the A-share and H-share markets. Investors should be wary of the A-H share market. After 2021, the range of CES300 Index yield volatility is narrowing, gradually converging to between −0.01 to 0.01, but there is still a volatile rebound trend. The stock index return forecast is the basis of market risk analysis. BPNN is used in A-H stock exchange market risk analysis to achieve high fitting accuracy, providing a way and a feasible algorithm for the A-H share exchange market risk analysis and improving the efficiency of market risk prediction. It is more effective, convenient, and accurate than traditional methods; BPNN has broad application prospects in such nonlinear fields.

The article "Risk Analysis of A-H Share Connect Market Based on Deep Learning and BP Neural Network" was published in 2022. Journal: Comput Intell Neurosci.

In parallel, due to the limitation of objective conditions, this study has the following shortcomings: since the CES300 Index was launched at the end of 2014, the experimental data are not sufficient, and larger sample size may fit a better predictive model. In addition, the influencing factors of market risk are complex, including politics, economy, and culture. The forecast indicators in this study mainly rely on micro-stock trading data and economic macro-indices but do not include political and cultural background factors. For example, in the context of the global pandemic, the impact of COVID-19 on stock market risks, and the impact of political factors such as trade frictions on the stock market may be factors that should be included in the indicator system in future research, and this issue needs to be improved in the next step.

## Figures and Tables

**Figure 1:** BP neural network structure.

**Figure 2:** The CES300 Index daily yield.

**Figure 3:** BP neural network structure topology.

**Figure 4:** Network training process.

**Figure 5:** Deep learning training error convergence process.

**Figure 6:** Training error distribution.

**Figure 7:** Goodness of fit.

**Figure 8:** Comparison of CES300 Index yield forecast and actual value.

**Table 1:** Market risk prediction indicator system (input layer node).

Dimension	No.	Indicator name	Indicator definition
Basic data	1	Opening price	Opening price relative to the index CES300
	2	Closing price	Closing price relative to the index CES300
	3	Highest price	Highest price in the day of the stock index CES300
	4	Lowest price	Lowest price in the day of the stock index CES300
	5	Trading volume	The total number of transactions of constituent stocks on a specified trading day
	6	Trading value	The total transaction amount of the constituent stocks on the specified trading day

Extended metrics	7	P/E (price-to-earnings ratio)	P/E (overall method) = (∑total market value)/∑net profit attributable to shareholders of the parent company
	8	P/B (price-to-book ratio)	P/B (overall method) = (∑ total market value)/(∑ net assets)
	9	Change rate of P/E	Change rate of price-to-earnings ratio
	10	Change rate of P/B	Change rate of price-to-book ratio
	11	Volatility 20 days	Last 20 days closing price volatility (equation (1)), *n* = 20
	12	Volatility 60 days	Last 60 days closing price volatility (equation (1)), *n* = 60
	13	Volatility 120 days	Last 120 days closing price volatility (equation (1)), *n* = 120
	14	Volatility 250 days	Last 250 days closing price volatility (equation (1)), *n* = 250
	15	BIAS	N-day BIAS = (the closing price of the stock market on the current day − N-day closing moving average) ÷ the N-day closing moving average (equation (2))
	16	MA	MA(N) = sum of N-day closing prices/N (equation (4))

Macroeconomic indicators	17	USD exchange rate	USD/CNY exchange rate on the trading day
	18	HKD exchange rate	HKD/CNY exchange rate on the trading day
	19	CPI (%)	Consumer price index, year on year (month)
	20	M2 (%)	Money and quasi-money supply, year on year (month)
	21	GDP (%)	Gross domestic product, fixed base period, quarter on quarter

*Note.* The data come from the iFIND database.

The article "Risk Analysis of A-H Share Connect Market Based on Deep Learning and BP Neural Network" was published in 2022. Journal: Comput Intell Neurosci.

**Table 2:** Training results.

Data set	Sample proportion (%)	Observations	MSE	R
Train	70	1220	1.1780e-05	0.9928
Validation	15	262	1.2718e-05	0.9539
Test	15	262	1.3881e-05	0.9429

## Data Availability

The data used to support the findings of this study are included within the article.
